This article has been retracted.

# Role of miR-498 Combined with CREB1 in Apoptosis and Invasion of Hepatoma Cell Line

**DOI:** 10.1155/2022/9621764

**Published:** 2022-02-24

**Authors:** Ming Zhu, Shan Gao, Xuefeng Ren

**Affiliations:** The First People's Hospital of Linping District, Hangzhou 311100, China

## Abstract

**Objective:**

To detect the expression levels of miR-498 in the hepatoma cells and to clarify the biological roles of miR-498 in hepatoma by investigating CREB1, which is the target of miR-498. This study provides a new biomarker for the early diagnosis and targeted therapies for hepatoma.

**Methods:**

The expression of miR-498 between hepatoma cells and hepatocytes was detected by qRT-PCR. miR-498 was overexpressed in hepatoma cells, and then, flow cytometry was used to analyze the cell apoptosis rate. Cell migration and invasion ability were evaluated by Transwell migration assay and Matrigel invasion assay. The downstream targets of miR-498 were searched in the biological database or related software, and the result can be verified by luciferase reporter assay. The knockdown of the downstream target using RNA interference detected its biological functions in hepatoma cells and was confirmed by cotransfection experiments.

**Results:**

miR-498 was downregulated in hepatoma cell lines compared with hepatocytes. The overexpression of miR-498 significantly promoted apoptosis. Luciferase reporter assays showed that miR-498 could target CREB1 3′UTR and CREB1 was one of the targets of miR-498. Knockdown of CREB1 also inhibited hepatoma cells' malignant potential and increased the apoptosis rate of hepatoma cells. CREB1 was able to alleviate the changes caused by miR-498 overexpression.

**Conclusions:**

miR-498 is downregulated in hepatoma cell lines. Therefore, miR-498 can be one of the potential molecular markers for hepatoma diagnosis. miR-498 plays a role in tumor suppression through regulating CREB1.

## 1. Introduction

Hepatocellular carcinoma is one of the most malignant tumors [1]. Hepatocellular carcinoma (HCC) is the most common primary liver cancer, accounting for about 85% of the total primary liver cancer. It is considered to be the second-highest cancer incidence rate in China. HCC mainly occurs in patients with chronic liver disease, accounting for 70-90% of the total HCC patients. Many clinical data showed that 50% of patients with hepatocellular carcinoma develop after being infected with the hepatitis B virus (HBV). At present, surgical resection, liver transplantation, radiotherapy, chemotherapy, interventional therapy, and molecular-targeted therapy are the first choice for treating liver cancer. However, due to the recurrence and metastasis of cancer cells, the long-term survival rate of liver cancer is not high. Therefore, effective diagnosis in the early stage of liver cancer is crucial [2–4].

MicroRNAs (miRNAs) are highly conserved and have a wide range of short nucleotide sequences of about 18-24 nt. The production and maturation of miRNAs require the participation of many proteins. MicroRNA usually regulates the expression of the gene by binding to the 3′end noncoding region (3′UTR) of the mRNA of its downstream target gene, which plays an important role in a variety of cell life activities. In addition, many studies have shown that miRNA is differentially expressed in tumor cells and their corresponding normal cells. It affects the biological characteristics of tumor cells by regulating a variety of specific target genes, which has a particular value in tumor diagnosis and treatment.

Through the study of the relevant data of liver cancer patients, we found that there are several miRNAs related to liver cancer, such as miR-26b [5], miR-214 [6], and miR-138 [7]. Many experiments have proved that miR-498 has different expressions in many kinds of tumors, such as breast cancer and lung adenocarcinoma. However, there is little research on miR-498 in liver cancer, and there is a lot of research space. CREB1 is a member of cyclic-AMP response element-binding protein (CREB), which is closely related to some miRNAs and plays an important role in the occurrence and development of some cancers [8–11]. In this study, the expression of miR-498 in hepatocellular carcinoma and its regulation on CREB1 revealed their role in the occurrence and development of hepatocellular carcinoma.

## 2. Materials and Methods

### 2.1. Materials and Reagents

The empty plasmid pcDNA3.0 and hepatoma cell line HepG2 were purchased from the Shanghai Institute of Biochemical Cells. The high glucose DMEM and fetal bovine serum (FBS) were purchased from the Gibco company, and Trizol reagent was purchased from Invitrogen. Dual-luciferase reporter kit and vector were from Promega company in the United States. Primary antibodies, such as rabbit polyclonal antibody of cyclic-AMP response element-binding protein 1 (CREB1), GAPDH monoclonal antibody, Bax monoclonal antibody, and Bcl-2 monoclonal antibody, were purchased from Abcam company. Secondary antibodies with HRP from corresponding species were purchased from the Li-COR company in the United States.

### 2.2. Plasmid Transfection

An appropriate number of cells in the logarithmic growth stage were inoculated on 6-well plates and cultured until the confluency was 40%-60% for transfection. To prepare transfection, 200 *μ*l serum-free plate, 12 *μ*l Lipo2000, 200 *μ*L serum-free medium, and 1.5 *μ*g plasmid mixture, mixtures are, respectively, mixed and placed at room temperature for 5 min. The mixture was vortexed again and set at room temperature for 20 min. The above dosage is one well in the 6-well plate, configured according to the number of wells in the actual experiment. The mixture was evenly transferred in each well.

### 2.3. Cell Culture

HepG2, HL-7702, and HEK-293T cells were cultured in high glucose DMEM. The working concentrations of fetal bovine serum and penicillin-streptomycin were 10% and 1%, respectively. The setting temperature of the cell incubator was 37°C, and the CO_2_ concentration was 5%. Cells are generally cultured until the cell density reaches 80%-90%, digested and dispersed with trypsin to the cell suspension, and then subcultured appropriately.

### 2.4. Total RNA Extraction and RT-qPCR

The total RNA of cells was extracted with reagent Trizol. After extraction, the quality of RNA was detected and quantified. Reverse transcription and real-time fluorescence quantitative polymerase chain reaction (qRT-PCR) were performed according to the relevant kit. If the expression of miR-498 is detected, the tailed miScript II RT Kit (Qiagen, Germany) is used for reverse transcription due to the short length of miRNA. If the mRNA expression was detected, the HiScript 1st Strand cDNA Synthesis Kit (Nanjing Nuovizan Biotechnology Co., Ltd.) was used for reverse transcription. miR-498 detection primer: F: 5′-CTTTCAAGCCAGGGGGC-3′, the corresponding downstream primer is self-contained in the tailing reverse transcription kit, which is universal; detection primer of CREB1 gene: CREB1-F: 5′-GTGTGTTACGTGGGGGAGAG-3′; CREB1-R: 5′-GCATCTCCACTCTGCTGGTT-3′.

### 2.5. Western Blot

The cells were collected in the Eppendorf Tube, and the cells were lysed with the appropriate intensity. Then, the protein was quantified by the BCA method to ensure that the protein equivalent was detected by electrophoresis. SDS-PAGE gel electrophoresis was applied and then transferred to the membrane, sealed, incubated with primary and secondary antibodies, and eventually developed. Among them, the blocking solution, primary antibody diluent, and secondary antibody diluent were all used related products of Biyuntian Company. The dilution ratio of primary antibody was 1 : 1000 and incubated overnight at 4°C, and the dilution ratio of secondary antibody was 1 : 5000 and incubated at room temperature for 1 h.

### 2.6. Luciferase Report Gene

The psiCHECK2TM plasmid containing the fragment of miR-498 target site on the 3′UTR of CREB1 was constructed and recorded as psiCHECK2TM-CREB1. HEK-293T cells were inoculated into 24-well plates and cultured to a density of 50%-60% for transfection. An appropriate amount of miR-498 mimics (synthesized in biological organisms) and psiCHECK2TM-CREB1 reporter gene plasmid were transfected into one well at the same time. The negative control groups were NC (attached with miRNA mimic synthesis) and psiCHECK2TM-CREB1. After 24 hours, the supernatant was removed, the cell particles were collected, and the cells were lysed with Passive Lysis Buffer. After centrifuging, 20 *μ*l supernatant was transferred into a 96-well whiteboard (mainly depending on the instrument reading the fluorescence value in the later stage). LAR II was actually added to detect fireflies' luciferase activity; then, Stop & Glo Reagent was added to inhibit the luciferase activity. Meanwhile, the luciferase activity of sea kidneys was detected simultaneously. The two fluorescence values are collected, counted, and calculated.

### 2.7. Matrigel Cell Invasion Assay

Matrigel matrix glue was prepared and laid on the upper chamber of the Transwell migration plate. After the tested cells were digested with trypsin, they were resuspended and inoculated with a serum-free culture medium in the upper migration chamber. They were placed in the cell incubator after adding the cell culture medium in the lower chamber. After 48 hours, cells were fixed with 4% paraformaldehyde for 15 minutes and stained with crystal violet for 5 minutes. The upper cells were wiped with a cotton swab, washed with PBS until the background was clear. Then, cells were placed in the oven for drying at 37°C, observed cells with the help of a microscope, and took pictures.

### 2.8. Transwell Cell Migration Assay

After plasmid transfection, the cells were digested and counted with trypsin, resuspended with serum-free culture medium, and placed in the upper migration chamber. A cell culture medium containing 10% fetal bovine serum in the lower chamber was added, and the plate was placed in the cell culture box for 24 hours, fixed with 4% paraformaldehyde for 15 minutes, and stained with crystal violet for 5 minutes. The upper cells were wiped off with a cotton swab, washed with PBS, and dried at 37°C. Take pictures with a microscope and count.

### 2.9. Apoptosis Experiment

The cells were digested with trypsin and centrifuged to the supernatant to obtain cell particles. The cells were resuspended with binding buffer, stained with Annexin Alexa Fluor 647 and Propidium Iodide (PI) at room temperature without light, and tested on the computer according to the operation instructions of flow cytometry, and the percentage of apoptotic cells was recorded.

### 2.10. Cell Scratch Test

After plasmid transfection, the cells were digested with trypsin and centrifuged to remove the supernatant to obtain cell precipitation. An appropriate number of cells were resuspended with a culture medium and laid in a six-well plate. The six-well plate was evenly crossed with a marker pen in advance. After the cells have adhered to the wall, the 10 *μ*l gun head shall draw a horizontal line perpendicular to the bottom plate of the six-well plate according to the straight line of the marker pen. The marked cells with PBS were washed, and the supernatant was removed. Supplement serum-free cell culture medium was added, and the plate was put into the incubator. Eventually, samples were collected and pictured at a fixed time.

### 2.11. Statistical Analysis

SPSS 22.0 was used to analyze the data, and the data were expressed as mean ± standard deviation. The independent samples *t*-test was used to compare the differences between the two groups, and *P* < 0.05 was considered statistically significant.

## 3. Results

### 3.1. Expression Level of miR-498 in Hepatocellular Carcinoma Tissues and Cells

qRT-PCR was used to detect the expression of miR-498 in a hepatoma cell line (HepG2) and normal hepatocytes (HL-7702) (Table 1). Compared with normal hepatocytes (HL-7702), the expression level of miR-498 in hepatoma cells (HepG2) was significantly different, and the expression level of miR-498 in hepatoma cells was lower (*P* < 0.001).

### 3.2. Role of miR-498 in Hepatocellular Carcinoma

To explore the role of differential miR-498 expression in hepatoma cells and normal hepatocytes, we transfected the plasmid with overexpression of miR-498 into HepG2. The results of qRT-PCR showed that the transfection was effective, and miR-498 was overexpressed in HepG2 (Figure 1(a)).

We further studied the relationship between miR-498 overexpression and hepatoma cell proliferation. Western blot was used to detect the expression of related proteins in cells after miR-498 overexpression. The results illustrated increased apoptosis-promoting gene Bax and decreased apoptosis inhibiting gene Bcl-2 when miR-498 was overexpressed (Figure 1(b)). Therefore, we speculate that overexpression of miR-498 mainly inhibits the proliferation of hepatoma cells by promoting apoptosis, thus affecting the proliferation of hepatoma cells.

Cell migration was detected by the cell scratch test. The results showed that the fusion rate of the miR-498 overexpression group was slightly lower (Figure 1(c)) compared with the NC group (EGFP), indicating that miR-498 can inhibit the migration and invasion of hepatoma cells.

### 3.3. CREB1 Is a Downstream Target Gene of miR-498

We searched the complementary mRNA of miR-498 on the base sequence in the database to explore the molecular mechanism of the role of miR-498 (Figure 2(a)). There is a potential target of miR-498 on the 3′UTR of cyclic-AMP response element-binding protein 1 (CREB1). A luciferase reporter gene experiment verified the prediction results. It was detected that the luciferase activity of the wild-type CREB1 3′UTR (WT) group transfected with miR-498 was lower than that of the mutant (MUT) group, and the luciferase activity of the mutant group had no effect on whether miR-498 was transfected or not (Figure 2(b)). In addition, Western blot results showed that protein expression of CREB1 also significantly decreased after HepG2 overexpressed miR-498 (Figures 2(c) and 2(d)). Based on the above results, a target region on CREB1 3′UTR can bind to miR-498. Furthermore, there is a negative correlation between miR-498 and CREB1 expression.

### 3.4. Effect of Knockdown of CREB1 on the Biological Function of Hepatoma Cells

Using the principle of RNA interference, we designed siCREB1 to be transfected into hepatoma cell line HepG2, knocked down CREB1. qRT-PCR was used to detect the expression level of CREB1 before and after HepG2 knockdown. The results showed that the expression of CREB1 significantly decreased transfection. Western blot demonstrated consistent results (Figures 3(a) and 3(b)). In addition, knockdown of CREB1 also reduced cell migration and invasion (Figure 3(c)).

The above results identified that CREB1 is a target gene downstream of miR-498. Meanwhile, CREB1 also has a certain impact on the biological characteristics of hepatoma cells. Therefore, it is speculated that miR-498 affects the biological characteristics of hepatoma cells through the regulation of CREB1. To verify this regulation, we transfected miR-498 and CREB1 into hepatoma cell HepG2 simultaneously (Figure 4(a)) to detect the changes of cell-related functions. The results showed that the apoptosis rate of cells in the miR-498 and CREB1 cotransfection group was higher than that in the miR-498 overexpression group. However, there was still a difference compared with the control group. Similarly, cells' ability in the miR-498 and CREB1 cotransfection group increased compared with the miR-498 overexpression group. However, there was still a difference compared with the control group (Figures 4(b) and 4(c)). The above results show that miR-498 affects the biological characteristics of hepatoma cell HepG2 by regulating CREB1, and CREB1 can alleviate the functional changes of hepatoma cells caused by miR-498 overexpression.

## 4. Discussion

Hepatocellular carcinoma (HCC) is a common malignant tumor, which seriously threatens human health. The 5-year survival rate of liver cancer patients worldwide is only 30%-40%, and even lower in some countries or regions. Due to the strong concealment in the early stage of liver cancer, most patients with liver cancer diagnosed clinically have been in the middle and late stages. Therefore, the treatment strategy poorly affects moderate and late liver cancer patients, resulting in poor prognosis and missing the best treatment period [2]. Therefore, there is an urgent need to diagnose early patients with liver cancer effectively. With the rapid development of biomedicine and related science, some effective molecular markers have been screened, but these molecular markers still have defects and deficiencies in sensitivity and specificity. Therefore, we need to find and screen molecular markers for the early diagnosis of liver cancer with higher sensitivity and specificity [4].

Mature miRNA exists in various human body cells and tissues and shows tissue specificity. Previous studies have found that many diseases such as hepatitis, liver fibrosis, and liver cancer are closely related to miRNA at the molecular level [7]. Particularly in liver cancer, such as miR-494 [8], miR-221 [9], miR-498 [10], and let-7c [11], and related lncRNAs also cooperate with miRNAs to participate in the occurrence and development of liver cancer [12–14]. Cyclic AMP response element-binding protein (CREB) is an important transcriptional regulatory protein. By identifying and binding DNA cAMP response element (CRE), CREB participates in and regulates gene transcription through autophosphorylation or nonphosphorylation under the action of protein kinase [15]. In recent years, researchers focused on the nervous system such as Parkinson's disease [16, 17] and depression. By comparing the expression of CREB in different pathological tissues, it is found that CREB may be involved in the occurrence and development of many tumors since CREB expression level and activity in leukemia [18], renal cell carcinoma [19], and esophageal cancer [20] are higher than those in normal tissue. At present, more than 10 CREB proteins have been found, among which the research on CREB1 is relatively extensive. Combined with various previous results, researchers found that CREB is an important protooncogene in the human body, and it is also closely related to miRNA. Whether the interaction between CREB and miRNA plays a vital role in liver cancer remains to be studied and found [21].

This study studied and discussed the effects of miR-498 and CREB1 on many biological behaviours of hepatoma cells during the occurrence and development of hepatoma. It was found that miR-498 had noticeable expression differences between hepatoma cells and normal hepatocytes, and it was a potential molecular marker for the early diagnosis of hepatoma. In addition, overexpression of miR-498 in hepatoma cells can significantly promote hepatoma cell apoptosis and inhibit its invasion. CREB1 is one of the downstream target genes of miR-498, which can play an anticancer role under the targeted regulation of miR-498. It was found that the knockdown of CREB1 in hepatoma cells could promote apoptosis and inhibit the migration and invasion of hepatoma cells. As the downstream target gene of miR-498, CREB1 is regulated by it, which affects the biological characteristics of hepatoma cells. CREB1 can alleviate the functional changes of hepatoma cells caused by miR-498 overexpression.

In this study, the effect of miR-498 on apoptosis, migration, and invasion of hepatoma cells by regulating CREB1 has only been confirmed in vitro. Animal experiments in vivo have not further clarified it. In addition, CREB1, as a crucial functional protein, affects the biological characteristics of hepatoma cells under the control of miR-498. Whether there are other effector proteins or mechanisms downstream of CREB1 remains explored.

## Figures and Tables

**Figure 1:** Effect of overexpression of miR-498 on biological characteristics of hepatoma cell Hep G2. (a) The transfection efficiency of miR-498 plasmid was detected by qRT-PCR; (b) Western blot was used to detect the expression of apoptosis promoting gene Bax and apoptosis inhibiting gene Bcl-2 after overexpression of miR-498; (c) the cell scratch test was used to detect the migration ability of HepG2 cells after overexpression of miR-498. ^∗∗∗^*P* < 0.001; NS: no significance.

**Figure 2:** CREB1 is the target gene of miR-498. (a) Possible binding sites of miR-498 and CREB1; (b) after constructing CREB1 3′UTR luciferase reporter plasmid and cotransfecting HepG2 cells with miR-498 mimics, the experimental results of luciferase reporter gene were obtained; (c) after overexpression of miR-498 in HepG2 cells, the expression level of CREB1 gene; (d) after overexpression of miR-498 in HepG2, the protein expression level of CREB1. ^∗∗∗^*P* < 0.001; NS: no significance.

**Figure 3:** Effect of knockdown of CREB1 on Hep G2 cells. (a) qRT-PCR was used to detect the expression level of CREB1 in cells after knockdown of CREB1; (b) Western blot was used to detect the expression level of CREB1 in cells after knockdown of CREB1; (c) Transwell test showed that the migration and invasion of cells decreased after knockdown of CREB1.

**Figure 4:** Effect of miR-498 regulating CREB1 on biological characteristics of hepatoma cells. (a) Compared with overexpression of miR-498, the expression levels of miR-498 and CREB1 were detected by qRT-PCR; (b) Transwell assay was used to detect the migration and invasion of cells after CO transfection of miR-498 and CREB1; (c) the apoptosis rate of cells after CO transfection of miR-498 and CREB1 was detected by flow cytometry.

**Table 1:** Expression of miR-498 in normal hepatocyte HL-7702 and hepatoma cell HepG2.

Cell line	Relative expression level of miR-498
HepG2	1.02 ± 0.04
HL-7702	0.22 ± 0.03
*t*	29.875
*P*	<0.001

## Data Availability

The data used to support the findings of this study are included within the article.
